The article "Characteristics and Trends in Unethical Pro-organizational Behavior Research in Business and Management: A Bibliometric Analysis" was retracted in 2025. Reasons: unreliable results or conclusions; a conflict of interest; concerns about the peer review; concerns about the citations.

# Characteristics and Trends in Unethical Pro-organizational Behavior Research in Business and Management: A Bibliometric Analysis

**DOI:** 10.3389/fpsyg.2022.877419

**Published:** 2022-06-13

**Authors:** Zhihong Li

**Affiliations:** ^1^School of Management, Lanzhou University, Lanzhou, China; ^2^Evidence-based Social Sciences Centre, School of Basic Medical Sciences, Lanzhou University, Lanzhou, China

**Keywords:** unethical pro-organizational behavior, trends, research topic, bibliometric analysis, knowledge mapping

## Abstract

Unethical pro-organizational behavior is one of the core factors that affect organizational development. Although enterprises and researchers have done a lot of work, a quantitative and systematic assessment of unethical pro-organizational behavior research is still lacking, this review conducts a bibliometric analysis to describe the characteristics and trends of unethical pro-organizational behavior research in business and management, such as publication trend analysis, co-citation analysis, keywords co-occurrence analysis, and citation burst analysis. The results show that 89 articles and 4,523 references from 49 journals contributed by 254 authors are identified. The number of publications has increased significantly since 2019. The China and United States are the most productive country. Umphress E and Yam C are the most influential authors. “Journal of Business Ethics and Frontiers in Psychology” are the most influential journal, 26 words in 516 keywords constitute the strongest set of terms available, Keyword co-occurrence analysis found ethical decision-making, the measurement, and impact of unethical pro-organizational behavior, the antecedents of ethical leadership are worthy and prospective potential trends. These findings provide a systematically, transparently, and visually reviewed the landscape and development process of unethical pro-organizational behavior research, which may help researchers and practitioners to understand unethical pro-organizational behavior in business management and provide a new perspective for future research.

## Introduction

Corporate unethical behaviors is a type of corporate behavior that violates generally accepted social and ethical standards, such as data falsification (McCrum, 2019), false advertising (Zaleski., 2017), and falsified performance (Hakim and Ewing, 2015), those behaviors have occurred frequently in recent years (Umphress et al., 2010; Johnson and Umphress, 2019; Tang et al., 2020), these unethical behaviors bring not only significant economic losses to companies (Gee and Button, 2019; Seuntjens et al., 2019), but also cause indelible damage to companies’ reputation and future development (Cohen et al., 2013; Kilduff et al., 2016; Lee et al., 2019). Therefore, more and more researchers pay attention to corporate ethics (Kohlberg, 1969; Rest, 1986; Turker, 2009; Umphress et al., 2010), employees’ unethical behavior is considered an essential factor affecting the construction of corporate ethics (Kohlberg, 1969; Rest, 1986; Tenbrunsel, 1998). Unethical behavior harms others, violates the law or general moral standards, such as cheating and data falsification (Kohlberg, 1969). Since then, scholars have studied individual factors, and organizational environments, such as managerial gender (Kavanagh, 1996), ethical outlook (Kish-Gephart et al., 2010), team moral climate (Kulik et al., 2008), ethical leadership (Mayer, 2010), organizational goals (Schweitzer and Douma, 2004), and corporate culture (Trevino et al., 1998). These studies reveal some driving factors and some characteristics of unethical behavior and enrich the understanding of the mechanism of unethical behavior.

The article "Characteristics and Trends in Unethical Pro-organizational Behavior Research in Business and Management: A Bibliometric Analysis" was retracted in 2025. Reasons: unreliable results or conclusions; a conflict of interest; concerns about the peer review; concerns about the citations.

Later, Umphress et al. (2010) noted that several positive organizational elements, for example, organizational support and charismatic leadership, could be drivers of unethical pro-organizational behavior (UPB), UPB refers to the behavior of an organization’s employees that is contrary to the core values, laws, or ethical standards of society in order to maintain the interests or the effective operation of the organization (Umphress et al., 2010), such as making false accounts (McCrum, 2019) and intentionally covering up product defects (Zaleski., 2017). The introduction of the concept of UPB deepened the traditional understanding of UPB, it thus has attracted the attention of many researchers and practitioners in the field of business management. For example, Du et al. (2016) summarized the general characteristics of UPB in the business field (Du et al., 2016). Ramachandran et al. (2020) outlined the pattern of employees’ unethical behavior during the past decades (Ramachandran et al., 2020). Coskun and Ulgen (2017) summarized the drivers and critical characteristics of UPB (Coskun and Ulgen, 2017), and Volkswagen Group developed whistleblower system to reduce employee’s unethical behavior so as to benefit their organization, whistleblower system is a system for timely reporting potential violations of employees (such as violation of laws and regulations, violation of codes of conduct, internal policies, and involving the development of potential or known cheating devices; Guardian, 2019; Volkswagen, 2022). These studies further enhance our understanding of UPB in the business management field.

While these articles provide insight into the current state of UPB research, they pay attention to a relatively narrow and specific segment, such as selecting some drivers and characteristics. Moreover, previous reviews rely on qualitative methods, and there is no bibliometric research in this field. With the emergence of many articles on UPB research, there is an urgent need to conduct an up-to-date review to comprehensively and systematically describe the characteristics and trends of unethical pro-organizational behavior research. Bibliometric analysis as a quantitative review method not only minimizes selection bias during the sampling process the sampling process and the analysis processes are both open and visible; it can provide a higher level, evidence-based visual review of integrity and reduces experimental time or range restrictions for scholars (VanEck and Waltman, 2010; Hota et al., 2020; Li et al., 2020; Verma and Gustafsson, 2020). Especially in recent years, more and more attention has been paid to bibliometric analysis. For example, Gupta et al. (2021) visualized the landscape and development of international entrepreneurship orientation through bibliometric research (Gupta et al., 2021). Ferasso et al. (2020) used bibliometric methods to investigate the association between circular economy and business models in the current business and management literature (Ferasso et al., 2020). Therefore, it is essential to conduct a systematized, quantified, clear, and visible overview of the development of UPB research.

The article "Characteristics and Trends in Unethical Pro-organizational Behavior Research in Business and Management: A Bibliometric Analysis" was retracted in 2025. Reasons: unreliable results or conclusions; a conflict of interest; concerns about the peer review; concerns about the citations.

Therefore, we analyzed 89 articles and 4,523 references through bibliometric analysis to systematically, transparently, and visually review the landscape and development process of UPB research. The paper is structured in the following ways:

1. The developmental trajectory of UPB research is described, including publication trends, most cited articles, most productive authors, most productive countries and institutions, and most influential journals,
2. We visually describe the development track and specific relevance of keywords through keyword analysis, which provides insight into the theoretical constructs of UPB research and helps identify current and future research areas (clusters),
3. A co-citation analysis of authors, journals, and references was constructed to visualize the network relationships among them, and
4. A citation burst analysis of concerns was conducted to explore the dynamic changes and new knowledge turning points in UPB research.

## Theoretical Background

### Conceptualization of UPB

Unethical pro-organizational behavior was initially introduced by Umphress et al. (2010) and is defined as intentional unethical behavior of employees use that violates society’s moral code but benefits the organization. It consists of two essential aspects:

1. It is immoral, violating the legal or widely acceptable ethical norms, and
2. It is beneficial to the nature of the organization, where such behavior that is not explicitly prescribed or ordered by superiors is beneficial to the organization.

The article "Characteristics and Trends in Unethical Pro-organizational Behavior Research in Business and Management: A Bibliometric Analysis" was retracted in 2025. Reasons: unreliable results or conclusions; a conflict of interest; concerns about the peer review; concerns about the citations.

Later, according to Umphress and Bingham (2011), unethical pro-organizational behaviors are intentional behaviors committed by individuals that contributes to productive operation or enables its members to perform productively while violating the society’s core values, ethical practices, laws, and norms of proper behavior. Meanwhile, it provides three boundary conditions for UPB:

1. The action should be on purpose and not due to mistakes, errors, or unconsciousness,
2. The basis for determining UPB is the beginning of the act and not the result, often the motivation for unethical behavior is aimed at the group or its employees, whether the result is good for the organization or not,
3. If the original purpose of such behavior is private gain, although the act is beneficial to the company or its employees simultaneously, it does not belong to UPB; that is, UPB is based on altruistic motivation. Since then, the definition has gradually become widely accepted.

### Structure and Measurement of UPB

Although some measures of unethical behavior have emerged, there is still no uniformity in the testing of UPB, and the emergence of these measures will contribute to the understanding of boundary conditions, causes, and outcomes of UPB.

The first of these is the six self-report measures approaches proposed by Umphress et al. (2010), which uses a 7 point Likert items using “1” to indicate strong disagreement and “7” to indicate strong agreement, the form of measurement is self-report, such as “When it makes my group work effectively, I will conceal insufficient data about the firm’s offerings.” The scale has seven items, while the factor loading of the last is relatively low, so it is (often) ignored by some researchers. The scale is often used domestically and internationally, which retains the first six-question items.

Later, Xia (2014) studied the causes and outcomes of UPB based on this scale; he pointed out the incompleteness of the one-dimensional structure and defined UPB as a two-dimensional structural concept based on pro-organization and altruism (Xia, 2014), pro-organizational dimension refers to unethical behavior that is good for the group and does not harm the group’s members. Among them, UPB is composed of both self-interest and selfless self-interest. This may include some cultural differences, and Asian countries, such as China, are more collectivist, while Western European and American countries are more individualistic (Hofstede, 1984; McSweeney, 2002). Some empirical research results show that many factors mediate and moderate UPB, such as individual and leadership levels. Wang et al. (2018) proposed that previous studies focused on individual behavior; UPB is individual and organizational behavior. Therefore, two levels of UPB were offered: (1) at the individual level, the spontaneous behavior of employees in violation of social ethics is to promote organizational operation efficiency (Wang et al., 2018). It is a bottom-up phenomenon when individuals commit UPB in the organization. The behavior will gradually spread and lead to UPB in the organization, and (2) the organizational level is a top-down phenomenon. However, the two levels of UPB raised have not been verified by their research (Wang et al., 2018).

The article "Characteristics and Trends in Unethical Pro-organizational Behavior Research in Business and Management: A Bibliometric Analysis" was retracted in 2025. Reasons: unreliable results or conclusions; a conflict of interest; concerns about the peer review; concerns about the citations.

## Materials and Methods

Systematic Bibliometric Analysis is widely used to track the knowledge connection in many research disciplines. It can identify new research hotspots and trends through the knowledge base of old literature and follow the characteristics of objectivity, system, replicability, openness, and transparency. It can also reduce the bias brought by humans or systems (Dabi et al., 2020; Li et al., 2021). The systematic bibliometric analysis follows the international standard process (see Figure 1; Page et al., 2021a) and provides detailed information on each step. Compared with the traditional retrospective review, systematic bibliometric analysis combines qualitative and quantitative methods to review the UPB studies, providing a new perspective for future practitioners and researchers.

**Figure 1:** UPB research search and selection process (Based on the PRISMA 2020 statement).

### Data Collection

The literature data was from Web of Science (WOS) database, which covers more disciplines and can provide more comprehensive text information for bibliometric analysis. First, before searching, we developed a pre-search strategy (mainly by keywords). After reviewing relevant articles, we used the following strategy to explore the WOS database under the guidance of an information retrieval specialist: TS = [(Unethical Pro-organizational Behavio*) OR (Pro organizational Unethical Behavio*) OR (Non ethical Pro-organizational Behavio*) OR (Pro-organizational Non ethical Behavio*)], with the time span from 1980 to 2021. “TS (Topics)” was chosen to obtain as many relevant publications as possible; the research area was “management OR business,” the language was restricted to “English,” and there is no limit to the type of document type, the searching was conducted at evidence-based management center in January 1, 2022. Second, two authors retrieved data independently from the WOS database and identified studies by checking titles, abstracts, keywords, and full text after removing duplicate articles. Records were exported as “plain text” and “full records and citations.” Any discrepancies in the extraction steps were discussed and/or resolved by experts. Standardized and suggested results were extracted, not limited to title, author, journal, citation count, publication year, affiliation, region, impact factor (IF), etc. (Li et al., 2020; Page et al., 2021b).

The article "Characteristics and Trends in Unethical Pro-organizational Behavior Research in Business and Management: A Bibliometric Analysis" was retracted in 2025. Reasons: unreliable results or conclusions; a conflict of interest; concerns about the peer review; concerns about the citations.

### Data Analysis

The collected data were analyzed in Microsoft Excel 2021, VOSviewer (Version 1.6.16), and CiteSpace (Version 5.8.R1). Microsoft Excel 2021 was used primarily for descriptive statistical analysis of the collected article data, such as author, journal of publication, year of publication, author organization, funding source, and so on. VOSviewer was used to map the co-occurrence network of authors, institutions, journals, and keywords, CiteSpace is used to generate the citation burst analysis of references.

## Results

Overall, the study covered 89 articles from 49 journals contributed by 254 authors between 1980 and 2021 (although only 2010 to 2021 were captured). These authors belong to 184 institutions in 23 countries, with 1,457 citations, with an average of 16.37 citations per year.

### Annual Trends in Number of Publications

Figure 2 shows the number and trend of papers published each year. UPB is a kind of immoral behavior. Although the construct of unethical behavior is already presented since 1991, the UPB research only began in 2010. The first research appeared in 2010, so 2010 became the starting of this study. The change in publications can be divided into two phases: the first stage is from 2010 to 2018, with an annual number of articles ranging from 1 to 6, with slow growth in the number of publications each year; the second stage is from 2019 to now, with more than 14 publications per year and a significant growth trend in the number of publications each year, which shows that since its introduction, UPB has been making continuous progress. According to the fitted trend line *y* = 0.5262e^0.3561x^ (*R*^2^ = 9,563) shows that the number of publications in 2022 will continuous growth. Therefore, the number of published articles of UPB research will maintain a fast growth trend.

**Figure 2:** Annual output of UPB research.

### Most Cited Articles

Table 1 shows the top ten papers with the most cited papers. Among the 89 UPB studies, total citations is 1,457, average citation per item is 16.37, among which three articles have more than 100 citations (3.4%), 30 articles have between 10 and 100 citations (33.7%), 28 papers have citations between 1 and 9 (31.5%), and 28 articles have 0 citations (31.5%). These highly cited papers provide a good reference for UPB research. However, this method still has limitations because the most cited papers do not always contribute the most, have the greatest impact, or are always the most relevant; for example, one of the reasons for these 28 articles that have not been cited is that they were all published in nearly 3 years (2019–2021), and there is a transitional period before the newly published articles are cited, and their potential value needs some time to be explored and validated, as the earliest concept of UPB (Umphress et al., 2010) proposed by Umphress et al. (2010) was only cited 2–8 times in the 4 years after its publication (2010–2013). Umphress and Bingham (2011) modified and improved the concept of UPB. In the 2 years after its publication, the number of citations was only once (2011–2012), after which their research was widely cited.

The article "Characteristics and Trends in Unethical Pro-organizational Behavior Research in Business and Management: A Bibliometric Analysis" was retracted in 2025. Reasons: unreliable results or conclusions; a conflict of interest; concerns about the peer review; concerns about the citations.

**Table 1:** The top 10 most cited articles in UPB research.

Rank	Title	Authors	Journal	Year	Total citations	Average per year
1	Unethical behavior in the name of the company: the moderating effect of organizational identification and positive reciprocity beliefs on unethical pro-organizational behavior	Umphress, E., Bingham, B., & Mitchell, S.	Journal of Applied Psychology	2010	278	23.17
2	When employees do bad things for good reasons: examining unethical pro-organizational behaviors	Umphress, E., & Bingham, B.	Organization Science	2011	217	19.73
3	The relationship between ethical leadership and unethical pro-organizational behavior: linear or curvilinear effects?	Miao, Q., Newman, A., Yu, J., & Xu, L.	Journal of Business Ethics	2013	100	11.11
4	Unethical for the sake of the group: risk of social exclusion and pro-group unethical behavior	Thau, S., Derfler-Rozin, R., Pitesa, M., Mitchell, S., & Pillutla, M.	Journal of Applied Psychology	2015	99	14.14
5	Relaxing moral reasoning to win: how organizational identification relates to unethical pro-organizational behavior	Chen, M., Chen, C., & Sheldon, J.	Journal of Applied Psychology	2016	91	15.17
6	Transformational leadership and follower's unethical behavior for the benefit of the company: a two-study investigation	Effelsberg, D., Solga, M., & Gurt, J.	Journal of Business Ethics	2014	90	11.25
7	Prosocial citizens without a moral compass? examining the relationship between machiavellianism and unethical pro-organizational behavior	Castille, M., Buckner, E., & Thoroughgood, N.	Journal of Business Ethics	2018	52	7.43
8	The effect of leadership style, framing, and promotion regulatory focus on unethical pro-organizational behavior	Graham, A., Ziegert, C., & Capitano, J.	Journal of Business Ethics	2015	51	12.75
9	Investigating When and Why Psychological Entitlement Predicts Unethical Pro-organizational Behavior	Lee, A., Schwarz, G., Legood, A., Greenwood, M., & Freeman, E.	Journal of Business Ethics	2019	44	14.67
10	Why and when does ethical leadership evoke unethical follower behavior?	Kalshoven, K., Dijk, V., & Boon, C.	Journal of Managerial Psychology	2016	41	6.83

Among the top 10 cited articles, the first one has the highest number of citations (278). This paper examines the association between organizational identity and UPB. Umphress et al. firstly proposed the concept of UPB (Umphress et al., 2010).

The article "Characteristics and Trends in Unethical Pro-organizational Behavior Research in Business and Management: A Bibliometric Analysis" was retracted in 2025. Reasons: unreliable results or conclusions; a conflict of interest; concerns about the peer review; concerns about the citations.

In the second paper, the number of citations is 217, ranking second. Umphress et al. Modified and improved the concept of UPB (Umphress and Bingham, 2011).

The third, the number of citations is 100. Miao et al. examined the upside-down U-shaped (curved) relationship on ethical leadership and UPB (Miao et al., 2013).

The fourth (99 citations) examines the impact of group UPB from a risk perspective (Thau et al., 2015).

The fifth (91 citations), from a social identity theory perspective and social cognitive theory, found that organizational identity can predict UPB (Chen et al., 2016).

The sixth (90 citations) found positively correlations between transformational leadership and employees’ intentions to participate in UPB (Effelsberg et al., 2014).

The seventh (52 citations), based on the trait activation theory, found that the dark trait of Machiavellism can make individuals more willing to participate in the UPB (Castille et al., 2018).

The eighth (51 citations) found that when leaders use the loss framework rather than the gain framework, inspiring and attractive transformational leaders produce a higher level of UPB than transactional leaders (Graham et al., 2015).

The ninth (44 citations) studies the mechanism of psychological rights in predicting UPB (Lee et al., 2019).

The tenth (41 citations) studies the deep connection mechanism between moral leadership and UPB (kalshoven et al., 2016).

### Most Productive Authors

Several 254 authors contributed to the UPB research; among them, two authors published three articles (0.8%), 27 authors published two articles (10.6%), and 225 authors published 1 article (88.6%). The top ten most productive authors are listed in Table 2, where Umphress E and Yam C are the most influential authors in this field with three publications each, Umphress E and his collaborator Bingham B opened the new area of UPB, followed by Bingham B, Cheng K, Effelsberg D, Gigol T, Graham A, He B, Zhang Y, and Liao Y, with two articles each. Among the top 10 most productive authors, four are from China, three from the United States, one from Singapore, one from Germany, and one from Poland. On the whole, few researchers are participating in the research of UPB, and the output is less. The most likely reason is that UPB has only developed for 10 years since its birth, and most of the articles and authors have been new in the past 3 years. This shows that the research of UPB is still in the “baby” stage, and will thrive in the future, and will gradually be concerned by more and more researchers, the contributions of 254 authors will lay a solid foundation for the further development of UPB.

The article "Characteristics and Trends in Unethical Pro-organizational Behavior Research in Business and Management: A Bibliometric Analysis" was retracted in 2025. Reasons: unreliable results or conclusions; a conflict of interest; concerns about the peer review; concerns about the citations.

**Table 2:** The top 10 most productive authors in UPB research.

Rank	Authors	Records	Organizations	Research interests	Total citations
1	Umphress E	3	University of Washington, United States	Strategic communications, negotiations, ethicalLeadership, organizational justice, ethicabehavior, and diversity	466
2	Yam C	3	National University of Singapore, Singapore	Behavioral ethics, leadership, and humor	32
3	Bingham B	2	Brigham Young University, United States	The interdependent and evolving exchangesamong employees, their organizations, and related external constituencies	448
4	Cheng K	2	Zhejiang University of Technology, China	Unethical pro organizational behavior, and altruistic behavior	25
5	Effelsberg D	2	Ruhr University Bochum, Germany	Unethical pro organizational behavior, leadership, and benefit	99
6	Gigol T	2	Warsaw School of Economics, Poland	Unethical pro organizational behavior, gender differences, and employee engagement behavior	11
7	Graham A	2	Suffolk University, United States	Egoistic norms, ethics, organizational identification, and unethical pro-organizational behavior	52
8	He B	2	Guangdong University of Technology, China	Organizational behavior and decision-making, cross-cultural human resource management, leadership model and development, and project management	6
9	Zhang Y	2	Guangdong University of Technology, China	Organizational behavior, and business ethics	6
10	Liao Y	2	Shanghai Normal University, China	Responsibility consciousness, service-oriented citizenship behavior, service-oriented leadership, and service performance	2

### Most Influential Journals

A total of 89 articles were published in 49 different journals, of which only one journal published more than ten articles (2%), 12 journals published between 2 and 7 articles (24.5%), and 36 journals published only one article (75.5%). Table 3 lists the top 10 most productive journals in UPB research, among which “Journal of Business Ethics” is the most influential journal, with 19 articles, the highest number of citations (484). The highest h-index (13), followed by “Frontiers in Psychology” with seven articles, 14 citations and an h-index of 2, “Journal of Applied Psychology” with four articles and 436 citations, and then followed by “Journal of Managerial Psychology,” “Personnel Review,” and “Leadership & Organization Development Journal, “all published three articles with 10–53 citations and an h-index of 1 or 2, and finally “Organizational Behavior and Human Decision Processes,” “Journal of Management,” “Management and Organization Review,” and “Social Behavior and Personality,” each with two articles, between 2 and 32 citations, and an h-index of 1 or 2.

The article "Characteristics and Trends in Unethical Pro-organizational Behavior Research in Business and Management: A Bibliometric Analysis" was retracted in 2025. Reasons: unreliable results or conclusions; a conflict of interest; concerns about the peer review; concerns about the citations.

**Table 3:** The top 10 Most influential journals in UPB research.

Rank	Journals	Records	% of 89	Average citations per year	H-index	Total citations	IF(5 years)
1	Journal of Business Ethics	19	21.348	25.47	13	484	5.453
2	Frontiers in Psychology	7	7.865	2	2	14	2.722
3	Journal of Applied Psychology	4	4.494	109	4	436	8.025
4	Journal of Managerial Psychology	3	3.371	17.67	2	53	2.619
5	Personnel Review	3	3.371	7.33	1	22	2.706
6	Leadership & Organization Development Journal	3	3.371	3.33	2	10	2.122
7	Organizational Behavior and Human Decision Processes	2	2.247	16	2	32	3.938
8	Journal of Management	2	2.247	6	1	12	11.818
9	Management and Organization Review	2	2.247	6	1	12	2.872
10	Social Behavior and Personality	2	2.247	1	1	2	0.959

H-index (h-index) is a novel method for evaluating academic achievement. It means that the given author/journal has published at least h papers that have each been cited at least h times, which reflects one author’s academic contribution.

### Most Productive Countries/Institutions

A total of 23 countries and 184 institutions participated in UPB research, with the majority of contributions coming from the United States and China (74/89, 83.1%), only two countries published more than ten articles (8.7%), 14 countries published between 2 and 9 articles (60.9%), and seven countries published only 1 article (30.4%). In terms of region, Asian countries were the most productive with 54 publications (54/89, 60.7%), followed by North America (35/89, 39.3%), Europe (20/89, 22.5%), and Oceania (9/89, 10.1%), Table 4 shows the top 10 most productive countries and institutions, and as far as the country is concerned, China was the most productive country with 41 publications (41/89, 46.1%), followed by the United States (United States) (35/89, 39.3%), and finally, Australia, England, Germany, Netherlands, South Korea, Pakistan, Singapore, and Canada with between 3 and 9 publications (16.6% in total). In terms of institutions, most were from China and the United States, with none publishing more than 10 UPB studies. The most productive was Tongji University from China with 5 UPB studies (5/89, 5.6%), followed by Shandong University (China), Shanghai Jiao Tong University (China), Texas A&M University, College Station (United States), The Texas A&M University System (United States), Drexel University (United States), Indian Institute of Management IIM System (India), National University of Singapore (Singapore), Shanghai Normal University (China), and University of Queensland (Australia) have published about 3–4 articles, while among the others, a total of 132 institutions published only 1 article.

The article "Characteristics and Trends in Unethical Pro-organizational Behavior Research in Business and Management: A Bibliometric Analysis" was retracted in 2025. Reasons: unreliable results or conclusions; a conflict of interest; concerns about the peer review; concerns about the citations.

**Table 4:** The top 10 most productive countries/institutions in UPB research.

Rank	Countries/Regions	Regions	Records	Organizations	Records
1	China	Asia	41	Tongji University (China)	5
2	United States	North America	35	Shandong University (China)	4
3	Australia	Oceania	9	Shanghai Jiao Tong University (China)	4
4	England	Europe	6	Texas A&M University, College Station (United States)	4
5	Germany	Europe	6	The Texas A&M University System (United States)	4
6	Netherlands	Europe	5	Drexel University (United States)	3
7	South Korea	Asia	5	Indian Institute of Management IIM System (India)	3
8	Pakistan	Asia	4	National University of Singapore (Singapore)	3
9	Singapore	Asia	4	Shanghai Normal University (China)	3
10	Canada	Europe	3	University of Queensland (Australia)	3

### Keywords Analysis

Keywords analysis is a specific association between words based on the number of keyword co-occurrences. It is used to determine the relationships between topics in the disciplines represented in this literature set, which in turn can assist in identifying areas (clusters) for current and future research that constitute the theoretical constructs or underlying themes of the research area (VanEck and Waltman, 2010; Nd et al., 2020).

To ensure the accuracy and completeness of the keyword classification of the articles, all keywords were chosen which includes the keywords provided by the authors (author keywords) and the supplementary keywords provided by web of science (keyword plus); in this way researchers can reduce the deviation and risk related to manual marking content and it is not easy to omit the potential key information provided in the article. It is very effective in investigating the knowledge structure of current and future scientific fields. In the implementation we set the keywords to appear at least seven times and finally 26 words in 516 keywords constitute the strongest set of terms available (Figure 3). The most important ten keywords are immoral pro organizational behavior (48) identification (37) performance (23) organizational identification (22) and model (21) moral discrimination (17) ethical decision-making (17) employees (16) transformational leadership (15) self (15).

The article "Characteristics and Trends in Unethical Pro-organizational Behavior Research in Business and Management: A Bibliometric Analysis" was retracted in 2025. Reasons: unreliable results or conclusions; a conflict of interest; concerns about the peer review; concerns about the citations.

**Figure 3:** Keywords co-occurrence network in UPB research.

From Figure 3, there are three clusters,

Cluster-1 (red) focuses on ethical decision-making, including 11 keywords. They are ineffective supervision, bad things, civic behavior, ethical decision-making, ethics, leader–member exchange, leadership, moral displacement, organizational identification, unethical behavior, work.

Cluster-2 (green) focuses on the measurement and impact of UPB, including 11 keywords. They are UPB, commitment, company, identification, modeling role, model, more identity, performance, self, transformational leadership, and medical role.

Cluster-3 (blue) focuses on the antecedents of ethical leadership, including four keywords. They are antecedents, employees, ethical leadership, and identity.

In this figure, keywords are color-coded according to frequency of occurrence and strength of association. The colors range from red (oldest year) to green and blue (most recent years). The UPB field has evolved from the previous focus on the oldest ethical decision-making topics to more specific and strategic topics, such as unethical pro-organizational behavior, leadership ethics, antecedents, performance, and other challenges that influence may present.

### Top Cited Authors’ Co-citation Networks

A number of 3,162 authors make up the co-citation network of authors in the UPB study. Based on the criterion of a minimum of 20 citations, 38 key authors were obtained, and their co-citation network was divided into three main clusters (Figure 4).

**Figure 4:** Co-citation network of the most cited authors in UPB research.

Cluster-1 (red) represents the formative stage of the UPB concept and is composed of 18 authors, among whom Aiken IS, Bass BM, Castille CM, Chen M, Graham KA, Kalshoven KA, Kong DT, Lee A, Matherne *CF*, Miao Q, Preacher KJ, Thau S, and Wang TL provide evidence for the systematic study of the formation and consequences of UPB in terms of the correlation between variables and UPB, Podsakoff PM, Kish-Gephart JJ, and Effelsberg D systematically studied the formation and consequence comparison of UPB by using systematic methods, such as meta-analysis, SEM method, and comparative method. Finally, Effelsberg D developed the concept of UPB based on them.

Cluster-2 (green) represents the developmental stage of UPB-related theories and models and consists of 10 authors, Bandura A in social learning theory and self-efficacy theory, Baumeister RF in computational social theory, and Tenbrunsel AE in ethical theory. They have contributed greatly to UPB-related theories and measurements. Trevino LK, Brown ME, Mayer DM, Detert JR, Gino F, Moore C, Reynolds SJ, and Tenbrusel AE focused on ethical models. They put forward the multi-level empirical model, effectiveness model, and immoral decision-making model of ethical leadership.

The article "Characteristics and Trends in Unethical Pro-organizational Behavior Research in Business and Management: A Bibliometric Analysis" was retracted in 2025. Reasons: unreliable results or conclusions; a conflict of interest; concerns about the peer review; concerns about the citations.

Cluster-3 (blue) represents the UPB decision-making process and its dual outcome impact and consists of 10 authors, Aquino K, Ashforth BE, Blau P, Cropanzano R, Eisenberger R, Greenberg J, Mael F, Mael F, Tajfel H, Van Knippenberg D focusing on unethical decision processes and dual outcome effects from different perspectives.

### Most Cited Journals

A total of 1,429 citations were obtained. We select the journals that published more than 30 articles so as to get the best co-citation relationship and make the results more appropriate. Finally, 30 journals meet the standard and are the most prominent in the co-citation relationship. These networks are mainly composed of five clusters (Figure 5).

**Figure 5:** Co-cited journals in UPB research.

Cluster 1 (green): focusing on the eight most influential international journals in the field of organizational psychology, it is committed to the study of ethics in organizations from the perspective of psychology, including:

The “Journal of Applied Psychology” emphasizes new knowledge and understanding in applied psychology to strengthen understanding of cognitive, motivational, emotional, and behavioral psychological phenomena in work and organizational settings.

The “Journal of Business and Psychology” focuses on industrial/organizational psychology, work psychology, human resource management, occupational psychology, organizational behavior, and vocational psychology.

The “Journal of Management” focuses on empirical and theoretical articles on the workplace, it covers aspects of business strategy and entrepreneurship, policy, organizational behavior, human resource management, organizational theory, and others.

The “Journal of Occupational and Organizational Psychology” focuses on improving people’s understanding of people and organizations at work through interdisciplinary knowledge and methods, including industry, organization, work, occupational and staff’s psychology, behavioral and recognition aspect of labor relations, the human factor, etc.

The “Journal of Organizational Behavior” focuses on empirical paper and a theoretical review of organizational behavior, focusing on the research and theory related to organizational behavior in analyzing individuals, groups, and organizations.

The “Journal of Vocal Behavior” focuses on career choice, career development, and job adjustment in the whole life cycle.

The article "Characteristics and Trends in Unethical Pro-organizational Behavior Research in Business and Management: A Bibliometric Analysis" was retracted in 2025. Reasons: unreliable results or conclusions; a conflict of interest; concerns about the peer review; concerns about the citations.

The “Leadership Quarterly” is committed to promoting the understanding of leadership from different perspectives.

The “Organizational Research Methods” mainly improve the research methods in organizational behavior through qualitative, quantitative, or mixed methods.

Cluster 2 (purple): it mainly includes four international most influential journals related to business ethics, management, and psychology, and is committed to providing high-quality original research and theoretical research, including:

The “Journal of Business Ethics” focuses on ethical aspects linked with business, bringing something new or different to its field.

The “Journal of Business Research” investigate a variety of business strategies, processes, and practices in true business contexts. Regularly assesses ongoing theoretical and empirical developments in purchaser behavior, financial, organizational change theory and behavior, as well as marketing, venture, insured, and global business.

The “Journal of Managerial Psychology” emphasizes on the social influence of management psychology and the wide application of psychological theory and practice in human resource management.

The “Business Ethics Quarterly” specializes in the theoretical and empirical research on business ethics, including the domestic ethics of business organizations, the role that business organizations play in the context of larger social, political, and cultural frameworks, and the ethical dimensions of market societies and the ethical quality of marketing relationship.

Cluster 3 (red face): focuses on the research of social psychology in organizations through experimental or non-experimental methods, and deepens the research of business ethics through the perspective of social psychology.

The “Annual Review of Psychology” focuses on the main development of psychology, including personality psychology, human development, community psychology, social psychology, environmental psychology, etc.

The “Journal of Experimental Social Psychology” focuses on using experimental or non-experimental methods to expand or create social psychology.

The “Journal of Personality and Social Psychology” focuses on psycho-social and psycho-social psychology.

The “Organizational Behavior and Human Decision Processes” concentrates on basic study of organized behavior, psychology, cognition, judgment, and decision taking of human beings.

The “Personality and Social Psychology Bullet” focuses on the field of personality and social psychology through original empirical research.

The “Personality and Social Psychology Review” focuses on theoretical papers and concept reviews in personality and social psychology.

The article "Characteristics and Trends in Unethical Pro-organizational Behavior Research in Business and Management: A Bibliometric Analysis" was retracted in 2025. Reasons: unreliable results or conclusions; a conflict of interest; concerns about the peer review; concerns about the citations.

The “Psychological Bullet” focuses on the evaluation and comprehensive research review and explanation of psychological problems, including qualitative (narrative) and/or quantitative (meta-analysis).

The “Psychological Science” specializes in the newest discoveries from cognitive, social, developmental, and wellness psychology to performance psychology and psychology of biology.

Cluster 4 (yellow): there are four kinds of magazines, mainly from the interpersonal relationship, personality structure, psychological data interpretation, to study the immoral behavior in the organization, as follows:

The “Human Relations” focuses on improving our understanding of our work and the social relationships around us. Interpersonal relationships encourage strong empirical contributions, develop and expand theories, and more conceptual papers integrate, criticize and expand existing theories.

The “Personal and Individual Differences” focuses on experimental, relevant, theoretical, explanatory/comprehensive research to enhance the understanding of personality structure and other forms of individual differences and the process leading to these individual differences and their practical application.

The “Personal Psychology” focuses on people-centered psychological research at work, including human resource management and organizational behavior.

The Psychological methods focus on developing and disseminating methods for analyzing, understanding, and interpreting psychological data.

Cluster 5 (blue): there are six kinds of magazines, which mainly study unethical behaviors in organizations from multiple methods, perspectives, and technologies.

The “Academy of Management Journal” focuses on testing, expanding, or establishing management theory through various research methods, and contributing to management practice, including providing original evidence for the study of UPB.

The “Academy of Management Review” focuses on different perspectives to promote understanding of management and organization. Administrative science quarterly focuses on the best theoretical and empirical research of organization research and interdisciplinary work of organization theory.

The “Journal of Marketing Research” focuses on the concepts, methods, and applications of marketing research.

The “Organization Science” focuses on the process, structure, and technology of organizational behavior.

The “Research in Organizational Behavior” focuses on research from persons to teams and then to institutions and their circumstances.

### Citation Burst Analysis of References

Burst analysis of citations can identify and track publications with strong citation growth characteristics. The surge means that an article has been cited quickly in the past few years, which marks the dynamic change of the research field and a new turning point of knowledge.

The article "Characteristics and Trends in Unethical Pro-organizational Behavior Research in Business and Management: A Bibliometric Analysis" was retracted in 2025. Reasons: unreliable results or conclusions; a conflict of interest; concerns about the peer review; concerns about the citations.

Figure 6 indicates that 13 references have the strongest citation bursts. Among them, Effelsberg D studied the ethical behavior of employees as a result of transformational leadership in 2014. Its new focus on learning the ethical dimensions of transformational leadership led to the most vigorous citation burst in this one between 2015 and 2019, with a burst intensity of 6.3, followed only by Umphress et al. (2010) and Umphress and Bingham (2011) on UPB concept with an outbreak intensity of 5.27, indicating the tremendous early attention given to UPB research by the scientific community.

**Figure 6:** Citation bursts analysis of references in UPB research.

In terms of the timing of the outbreak, Graham et al. (2015) and Thau et al. (2015) continue to explode from 2018 to 2019, respectively, which are the latest outbreaks of citations. Graham et al. (2015) addresses the implications of promotion control and leadership on staff intentions to perform UPB.

Thau et al. (2015) explores how being excluded from risk from the group motivates group members to involve in unethical behaviors that lead to better outcomes for the group, which provides a theoretical mechanism explanation for when and why UPB occur; thus, the issue of theoretical mechanisms of UPB could become a new turning point and hold great promise for UPB research in the coming years.

## Discussion

This paper discusses the knowledge structure and evolution of UPB research by using bibliometrics. Firstly, this paper expounds on the development track of the study on UPB, including the publishing trend of publications, the most cited articles, the most productive authors, the most productive countries and institutions, and the most influential journals. Second, the trajectory and specific associations of keywords are vividly described by keyword analysis, which provides an understanding of the theoretical construction of UPB research and identifies areas (clusters) for current and future research. It provides help to understand the theoretical construction of UPB research and identify areas (clusters) for the draft and future research. Third, a co-citation analysis of authors, journals, and references is constructed to reflect the network relationships among them graphically. Fourth, a citation burst analysis of concerns was conducted to explore the dynamic changes and new knowledge turning points in UPB research.

### Theory Significance and Future Research Trends

The work has made some theoretical references to the UPB. First of all, we contributed to UPB research and quantitatively mapped the publications of UPB research. In Figure 2, UPB research has been gaining more interest from researchers in recent years, especially in the past 3 years. The number of publications on UPB research has shown a double-digit growth trend. However, by investigating the research directions, we found that the number of published articles varies greatly, such as Business Economics with 65 publications and Psychology with 33 publications.

The article "Characteristics and Trends in Unethical Pro-organizational Behavior Research in Business and Management: A Bibliometric Analysis" was retracted in 2025. Reasons: unreliable results or conclusions; a conflict of interest; concerns about the peer review; concerns about the citations.

In contrast, other directions account for a tiny percentage. One reason for this unbalanced state may be the different perspectives, experimental designs, and research on various trends of UPB. Therefore, for the growing field of UPB, it is crucial to periodically review and assess its evolutionary pathways (Kohlberg, 1969; Rest, 1986; Verk et al., 2019), and we would like to inspire future researchers to enhance interdisciplinary synthesis to promote and coordinate the evolution of UPB research.

Second, although UPB has been widely studied in business research, the publication is of low quality. We find that although many articles have been published in business management, applied psychology, social psychology, labor relations, and other fields, the proportion of papers published in top journals (such as 4* journals, UTD24, or FT50) in these fields is small (less than 10%), UPB is very popular in these fields. However, the number of publications in the psychological field (applied psychology and social psychology) is far lower than that in business management. Therefore, future researchers need to strengthen the theoretical basis, experimental design, and data analysis (Ramachandran et al., 2020; Yan et al., 2020; Mishra et al., 2021), such as in the case of UPB research, an argument could be made that less theory-based and experimental research needs to be done, and more research needs to be done on measuring the effects of UPB, in terms of economic losses, damage to companies’ reputation and future development, harm to others or to general moral standards.

Third, our quantitative analysis helps to know the comparative contribution of individual countries and institutions to UPB research, with China and the United States contributing the most to UPB research, with no single institution publishing more than 10 UPB studies, and the most productive institution being Tongji University from China. However, our country/institution collaboration analysis revealed that there are few collaborative network relationships between countries and institutions, suggesting that UPB development is not equal across countries/institutions; therefore, we encourage research collaboration across institutional and national boundaries to discover differences between UPB studies and thus promote UPB research.

The article "Characteristics and Trends in Unethical Pro-organizational Behavior Research in Business and Management: A Bibliometric Analysis" was retracted in 2025. Reasons: unreliable results or conclusions; a conflict of interest; concerns about the peer review; concerns about the citations.

Fourth, keyword co-occurrence analysis can better trace the development trend of UPB research and provide directional guidance for future research (Ivanov et al., 2020), contributing to the theoretical development of UPB. By analyzing the evolution of UPB keywords, we found that the keywords “unethical pro-organizational behavior,” “identification,” and “performance.” Keywords (e.g., “unethical pro-organizational behavior,” “identification,” or “performance”) have continued a steady and growing trend over time. This suggests that such themes still have excellent research potential and significance in future studies. Further, we have identified several emerging research topics recently, for example, “models,” “antecedents,” and “ethical leadership,” that capture novel and underlying trends in UPB research. Therefore, such worthy and prospective subjects could be of great interest to a more significant number of fellows and performers and contribute to our understanding of UPB research.

Fifth, we describe the relative contributions of authors, journals, and references in UPB research and the network relationships among them through citation analysis. Our author co-citation analysis found, for example, that the most substantial impact authors in the UPB study were Umphress E, Trevino K, and Ashforth E and other researchers and practitioners at different stages of research (e.g., Effelsberg D, Podsakoff M, Tajfel H, etc.) also made significant contributions to the development of UPB. The co-citation analysis of journals shows that the most influential journal for UPB research is the Journal of Applied Psychology. In addition, the citation burst analysis of references shows that the most bursting connection is Effelsberg D’s 2014 publication on the impact of transformational leadership on employees’ ethical behavior over time. Different researchers have also contributed, the most recent being Graham A and Thau S, who have examined the theoretical mechanisms of when and why UPB occurs and is still in a continuous burst phase, and these studies will contribute to the development of ethical development theory (Kohlberg, 1969) and ethical model theory (Rest, 1986). Therefore, UPB’s theoretical development and mechanism will be a new turning point and a promising development for UPB research in the coming years.

This study has a few insights for practitioners as well. To start with, our work contributed to practitioners’ thorough knowledge of the findings of UPB research in business management, which not only guides business management practitioners in managing employees and improving organizational performance but also contributes to its application in the field of psychology. Second, our study quantifies and visualizes leading-edge topics and the latest findings in UPB research. Researchers have found that UPB research is rapidly a frontier of commercial difference for companies, which may help leaders involved in business practices deal with UPBs of their employees or those in their organizations, thus improving employee output organizational performance. Third, country and institutional analyses aid practitioners get a comprehensive insight into UPB research in a global context, which may provide a potential competitive advantage for business management implementers.

The article "Characteristics and Trends in Unethical Pro-organizational Behavior Research in Business and Management: A Bibliometric Analysis" was retracted in 2025. Reasons: unreliable results or conclusions; a conflict of interest; concerns about the peer review; concerns about the citations.

## Limitations

Even though the bibliometric approach is powerful, some limitations need to be acknowledged. To begin with, whereas Web of Science is among the most widely used databases for visible research, it is not the source of the entire UPB research literature; therefore, our findings are limited by the WOS database, and we cannot exclude the possibility some of the data are missing. If the visualization technology matures in the future, we encourage collecting as many publications as possible to improve our study. Second, we only focus on UPB research in the business management field. However, UPB research is a worldwide disseminated theme that may also exist in, for example, medicine or the environment. Hence, future research needs to expand the scope of the study, which may help shed some light on the literature from other fields beyond business. Third, unlike traditional literature reviews which examine the research that has been done and tries to analyze/summarize/synthesize the meaning of the research, a Systematic Bibliometric Analysis only looks at the productions and citations (by county, by journal, by author) not their content, we did not examine the underlying connections of these relationships in detail, so further work could add to their deeper collaborative relationships.

## Conclusion

In contrast to classic reviews, this work proposes an updated bibliometric study to facilitate the trajectory of UPB research in business management. Specifically, by using Vosviewer and CiteSpace, we performed some crucial bibliometric analysis, consisting of publication mapping analysis, co-citation analysis, keywords co-occurrence analysis, and citation burst analysis, and we map the knowledge structure of UPB research in commerce management and capture its developmental path along time. Furthermore, we map the knowledge structure of UPB research in commerce management and capture its developmental way over time. Moreover, we propose several themes for further study based on our results. The work promotes a systematic and thorough insight into UPB research by conducting a bibliometric analysis of current knowledge structures and research trends and predicting future trends in UPB research.

The article "Characteristics and Trends in Unethical Pro-organizational Behavior Research in Business and Management: A Bibliometric Analysis" was retracted in 2025. Reasons: unreliable results or conclusions; a conflict of interest; concerns about the peer review; concerns about the citations.

## Data Availability Statement

The original contributions presented in the study are included in the article/supplementary material, further inquiries can be directed to the corresponding author.

## Author Contributions

The author confirms being the sole contributor of this work and has approved it for publication.

## Funding

This work was supported by the Major projects of NSFC: Big data-driven study of public safety risks in cities (grant no. 16JZD023), and Theoretical system, international experience and Chinese path of evidence-based Social Sciences (grant no. 19ZDA142).

## Conflict of Interest

The author declares that the research was conducted in the absence of any commercial or financial relationships that could be construed as a potential conflict of interest.

## Publisher’s Note

All claims expressed in this article are solely those of the authors and do not necessarily represent those of their affiliated organizations, or those of the publisher, the editors and the reviewers. Any product that may be evaluated in this article, or claim that may be made by its manufacturer, is not guaranteed or endorsed by the publisher.
